RETRACTED

# Hsa_circRNA_0008028 Deficiency Ameliorates High Glucose-Induced Proliferation, Calcification, and Autophagy of Vascular Smooth Muscle Cells via miR-182-5p/TRIB3 Axis

**DOI:** 10.1155/2022/5142381

**Published:** 2022-08-24

**Authors:** Lili Shi, Yuliang Li, Meixin Shi, Xiaoxue Li, Guopeng Li, Jie Cen, Dan Liu, Can Wei, Yan Lin

**Affiliations:** ^1^Department of Cadre Ward, The First Affiliated Hospital of Harbin Medical University, Harbin 150081, China; ^2^Department of Anesthesiology, The Fifth Hospital of Harbin, Harbin 150081, China; ^3^Department of Pathophysiology, Harbin Medical University, Harbin 150086, China; ^4^Department of Cadre Ward, The Fourth Affiliated Hospital of Harbin Medical University, Harbin 150081, China; ^5^Department of Pathophysiology, Qiqihar Medical University, Qiqihar 161006, China

## Abstract

**Background:**

It is well-known that dysfunctions of vascular smooth muscle cells (VSMCs) act an essential part in vascular complications of diabetes. Studies have shown that circular RNAs (circRNAs) and microRNAs (miRNAs) play a crucial role in regulating cell functions. However, their influence on the proliferation, calcification, and autophagy of VSMCs remains to be further explored. Therefore, this study elucidates the role and mechanism of hsa_circRNA_0008028 in high glucose- (HG-, 30 mM) treated VSMCs in *vitro*.

**Methods:**

Quantitative real-time polymerase chain reaction (qRT-PCR) was chosen to detect the levels of hsa_circRNA_0008028, miR-182-5p, and tribble 3 (TRIB3). Then, dual-luciferase reporter and RNA immunoprecipitation (RIP) assays were used to predict and verify the binding relationship between miR-182-5p and hsa_circRNA_0008028 or TRIB3. Cell counting kit-8 assay, 5-ethynyl-2′-deoxyuridine (EdU) staining, corresponding commercial kits, and western blotting were used to measure indexes reflecting cell viability, proliferation, calcification, and autophagy of VSMCs, respectively.

**Results:**

In HG-induced VSMCs, hsa_circRNA_0008028 and TRIB3 were highly expressed, whereas miR-182-5p decreased. Meanwhile, cell proliferation, calcification, and autophagy could be repressed by silencing of hsa_circRNA_0008028. However, these effects can be eliminated by miR-182-5p inhibition. Furthermore, it was demonstrated that hsa_circRNA_0008028 could promote the expression of TRIB3, a target of miR-182-5p, by directly sponging miR-182-5p. The expression of TRIB3 was suppressed by hsa_circRNA_0008028 knockout, which was rescued by miR-182-5p inhibition.

**Conclusion:**

This study reveals that hsa_circRNA_0008028 can act as a sponge of miR-182-5p and promote HG-induced proliferation, calcification, and autophagy of VSMCs partly by regulating TRIB3.

RETRACTED

## 1. Introduction

Diabetes, a multifactorial metabolic disorder, features hyperglycemia caused by absolute or relative lack of insulin secretion. Its related vascular diseases, especially microvascular ones, play a major influencing role in the prognosis and mortality of diabetic patients [1]. As known to all, VSMCs serve as the main component of the middle layer of the artery and show phenotypic plasticity as they can differentiate from a contractile/nonproliferating phenotype to a synthetic/proliferating one during vascular injury [2, 3]. Scholars said that diabetes or HG exposure might cause excessive proliferation and migration of VSMCs, further lead to calcification and vascular remodeling and promote diabetes-correlated vasculopathy [4, 5]. Therefore, inhibiting the dysfunctions of VSMCs such as abnormal proliferation, migration, and calcification may serve as a potential intervention target for diabetes-related vascular diseases.

circRNAs, a subfamily of noncoding RNAs, with multiple functions as reported, can act as the miRNA sponge or competing endogenous RNA (ceRNA) and compete for miRNA pairing with other RNAs [5–7]. It was reported that miRNAs could exert cellular functions by regulating the translation or stability of target mRNAs like cell growth, proliferation, differentiation, metabolism, immunity, and cell death [8–11]. The precise molecular and biochemical function of the majority of circRNAs and miRNAs remains unclear, but their roles in the functional regulation of VSMCs have been widely reported [2, 12, 13]. Over these years, circRNA LRP6, circRNA-0077930, and circWDR77, as well as miR-217, miR-381-3p, and miR-132 have been found to get involved in the HG-induced proliferation and migration of VSMCs [2, 14–18]. However, it remains unclear whether hsa_circRNA_0008028 and miR-182-5p perform biological functions in diabetes-correlated vasculopathy.

Studies showed that TRIB3 played a critical role in the induction and maintenance of contractile phenotype in VSMCs, and its expression suppression can inhibit vascular remodeling of VSMCs [19, 20]. However, the exact regulating mechanism remains unknown. Thus, this study is aimed at further exploring the underlying roles and molecular mechanisms of hsa_circRNA_0008028/miR-182-5p/TRIB3 in abnormal proliferation, calcification, and autophagy of VSMCs under HG exposure, and it is expected to discover potential therapeutic targets for diabetic vascular remodeling.

## 2. Materials and Methods

### 2.1. Cell Culture, Transfection, and Treatment

Human aortic vascular smooth muscle cells (ATCC, CRL-1999) were cultured in the Dulbecco's Modified Eagle's Medium (DMEM, HyClone, USA) supplemented with 10% fetal bovine serum (FBS, Gibco, USA), penicillin (100 U/mL, Beyotime, China), and streptomycin (0.1 mg/mL, Beyotime, China) in a humidified atmosphere with 5% CO_2_ at 37°C. Before the subsequent experiments, all cells were kept quiescent by starvation for 24 hours and then treated with 5.5 mmol/L D-glucose (normal glucose (NG)) or 30 mmol/L D-glucose (HG) for 48 hours. All VSMCs to be tested for calcification and osteogenic differentiation were treated with HG and coincubated with 10 mmol/L *β*-glycerophosphate (*β*-GP, Sigma-Aldrich, USA) for 12 days after siRNA transfection or overexpression [21]. VSMCs exposed to 30 mmol/L mannitol (MA, Aladdin, China) was chosen as the negative control.

RETRACTED

For cell transfection, VSMCs were transfected with hsa_circ_0008028 and TRIB3 siRNA, miR-182-5p mimic, and miR-182-5p inhibitor, while their corresponding negative control was treated using Lipofectamine 2000 (Invitrogen, USA). The siRNA targeting hsa_circ_0008028 (F: 5′-GAUUUCCCAGAUUCCUUUGUU, R: 5′-AACAAAGGAAUCUGGGAAAUC) was used to knockout hsa_circ_0008028, and siRNA negative control (si-NC) was used as a control. Moreover, miR-NC, miR-182-5p mimic, and miR-182-5p inhibitors were used to upregulate or downregulate its expression. All the plasmids were provided by GenePharma (Shanghai, China). The transfection effect was detected by qRT-PCR.

### 2.2. Cell Viability Assay

A quantitative evaluation of cell viability was performed by a Cell Counting Kit-8 assay (CCK-8, MedChemExpress, China). VSMCs were plated into 96-well plates at a density of 2 × 10^3^ cells/well added with10 *μ*L CCK-8 solution and incubated in the dark for 2 hours at 37°C. The absorbance at 450 nm was detected spectrophotometrically.

### 2.3. EdU Staining

A 5-ethynyl-2′-deoxyuridine (EdU) kit (RiboBio, Guangzhou, China) was used to detect cell proliferation. VSMCs were seeded in 96-well plates, incubated with EdU (50 *μ*mol/L) for 24 hours at 37°C, then washed with PBS, fixed in 4% formaldehyde for 10 minutes, stained with Apollo staining solution (100 *μ*L/well) for 30 minutes, and then stained with DAPI for 10 minutes at room temperature. All images were taken with a fluorescence microscope (BX61; Olympus, Tokyo, Japan). Fields were randomly chosen from three dishes, three for each, at least from each group to determine the number of EdU-positive cells.

### 2.4. Detection of Alkaline Phosphatase (ALP) Activity

After being washed with PBS twice, VSMCs' layers were scraped into a solution. The cell lysates were homogenized and measured for ALP activity by a commercial kit (Jian Cheng Bioengineering Institute, Nanjing, China) according to the manufacturer's instructions. As previously described, ALP activity was normalized to the total cellular protein of the cell layers by the Bradford protein assay [22].

RETRACTED

### 2.5. Dual-Luciferase Reporter Assay

The sequences of hsa_circ_0008028 and TRIB3 3′UTR, harboring the miR-182-5p seed region or a mutant sequence, were subcloned into the pmirGLO luciferase vectors (Promega, USA), referred to as WT-hsa_circ_0008028, MUT-hsa_circ_0008028, WT-TRIB3 3′UTR, or MUT-TRIB3 3′UTR, respectively. VSMCs were cotransfected with reporter plasmids and miR-182-5p mimic or miR-NC using Lipofectamine 2000. After 48 hours of transfection, the luciferase activities were tested by the Dual-Luciferase Reporter Assay System (Promega, USA).

### 2.6. RNA Immunoprecipitation (RIP)

RIP assays were performed by RNA-Binding Protein Immunoprecipitation Kit (Millipore, USA). VMSC lysates were incubated with RIP buffer containing magnetic beads conjugated with anti-Argonaute-2 (Ago2) or anti-immunoglobulin G (IgG) antibodies. After being purified, immunoprecipitated RNA was examined by qRT-PCR.

### 2.7. Western Blotting

The proteins in VSMCs were extracted separately and quantified using a BCA protein assay kit (Beyotime, China). Equal amounts of protein samples were separated by SDS-PAGE and electrotransferred onto a PVDF membrane (Millipore, Schwalbach, Germany). The membranes were incubated overnight with primary antibodies (at a 1 : 1000 dilution, 4°C) purchased from Cell Signaling Technology (Danvers, MA, USA) and Proteintech (Wuhan, China). Subsequently, the secondary antibody (ZSGB-BIO, Beijing, China) was added to the membrane and kept for 2 hours at room temperature. An enhanced chemiluminescent (ECL) kit (HaiGene, Harbin, China) and a multiplex fluorescent imaging system (ProteinSimple, California, USA) were chosen to detect these signals. The Bio-Rad Quantity One software (Bio-Rad Laboratories, Hercules, USA) was used to quantify and normalize the intensities of protein bands into GAPDH.

### 2.8. Quantitative Real-Time PCR (qRT-PCR)

Total RNAs were extracted from VSMCs using TRIzol reagent (Thermo Fisher Scientific, USA) and reversely transcripted into cDNA using a cDNA kit (Bimake, Houston, TX, USA) according to manufacturers' instructions. qRT-PCR was performed by SYBR Green qPCR Master Mix with an ABI PRISM® 7500 Sequence Detection System. U6 or glyceraldehyde 3-phosphate dehydrogenase (GAPDH) was regarded as the internal reference. Relative quantification was conducted using the 2^−∆∆CT^ method. The sequences of primers are shown in Supplementary Table (Table S1).

### 2.9. Statistical Analysis

All data were represented as the mean ± standard deviation (SD). SPSS 22.0 (IBM Corporation, USA) and GraphPad Prism 6.0 (GraphPad Software, USA) were chosen for data analysis and visualization, while paired or unpaired *t*-tests or one-way ANOVA was used for data comparison, followed by Bonferroni post hoc test. A *p* < 0.05 was indicated statistically significant.

RETRACTED

## 3. Results

### 3.1. hsa_circRNA_0008028 Is Highly Expressed in HG-Treated VSMCs

To investigate the functional role of hsa_circRNA_0008028 in VSMCs under HG conditions, qRT-PCR was used to evaluate its expression pattern. First, using mannitol (MA, 30 mmol/L) as the negative control, VSMCs were exposed to different concentrations of D-glucose (5.5, 10, 20, and 30 mmol/L). The results showed that the expression level of hsa_circRNA_0008028 rose with the increase in D-glucose concentrations but was not affected by MA stimulation (Figure 1(a)). Then, the results showed an upregulation of hsa_circ_0008028 expression in a time-dependent manner under D-glucose (30 mmol/L) incubation (Figure 1(b)). In the subsequent experiments, D-glucose at 30 mmol/L for 48 hours was selected as an HG condition. Thereafter, RNase R digestion was performed to verify the circular nature of hsa_circRNA_0008028. Results showed that RNase R^+^ lowered the mRNA level of GAPDH and had little effect on hsa_circRNA_0008028 expression (Figure 1(c)), suggesting that hsa_circRNA_0008028 was a circular and stable transcript resistant to treatment with RNase R digestion.

### 3.2. Silencing hsa_circRNA_0008028 Inhibits HG-Induced Proliferation, Calcification, and Autophagy of VSMCs

Given that hsa_circRNA_0008028 was highly expressed in HG-treated VSMCs, we knocked it down. The qRT-PCR results showed that si-hsa_circRNA_0008028 transfection significantly inhibited the HG-mediated upregulation of its expression compared with the siRNA negative control (si-NC) group (Figure 2(a)). The data of CCK-8 manifested that HG treatment enhanced the viability of cells, which was then notably reversed by knockdown of hsa_circRNA_0008028 (Figure 2(b)). Meanwhile, EdU assay and western blotting verified that si-hsa_circRNA_0008028 reduced HG-evoked cell proliferation and cyclin D1 expression in VSMCs (Figures 2(c), 2(d), and 2(f)).

To further verify the effect of hsa_circRNA_0008028 on cell calcification and osteogenic differentiation, HG-treated VSMCs were coincubated with 10 mmol/L *β*-glycerophosphate (*β*-GP) for 12 days after transfection [21]. As expected, obvious calcification, characterized by increased alkaline phosphatase (ALP) activity (Figure 2(e)) can be observed in cells in the HG group and the HG and si-NC group. Western blotting showed that HG increased the protein expression of osteogenic differentiation-related indexes including runt-related factor 2 (Runx2) and osteopontin (OPN) in VSMCs together with *β*-GP, whereas inhibiting the expression of SM *α*-actin (*α*-SMA) (Figure 2(f)). The above changes were notably mitigated by si-hsa_circRNA_0008028 transfection in VSMCs (Figures 2(e) and 2(f)), suggesting the inhibiting role of hsa_circRNA_0008028 silencing in the calcification and osteogenic differentiation in HG-induced VSMCs.

RETRACTED

Substantial evidence suggests that autophagy gets involved in the regulation of VSMCs disorder [4, 23]. We found that autophagy was activated in HG-stimulated VSMCs, shown as an increased LC3B-II/-I ratio and a decreased SQSTM1/p62 expression, which was abrogated by si-hsa_circRNA_0008028 (Figure 2(g)). To sum up, the above results showed that hsa_circRNA_0008028 interference could inhibit HG-induced proliferation, calcification, and autophagy of VSMCs.

### 3.3. hsa_circRNA_0008028 Binds to miR-182-5p

It was reported that circRNAs could regulate gene expression by binding to miRNAs as a sponge [24]. The starBase software was used to predict the potential binding sites between hsa_circRNA_0008028 and miR-182-5p (Figure 3(a)), which was later confirmed by dual luciferase reporter assay, as miR-182-5p overexpression markedly weakened the luciferase activity of wild-type (WT) hsa_circ_0008028 reporter rather than the mutated (Mut) hsa_circ_0008028 reporter (Figure 3(b)). RIP assay also verified the mutual effect of hsa_circ_0008028 and miR-182-5p at the endogenous level. Results showed that, compared to the control anti-IgG group (Figure 3(c)), hsa_circ_0008028 and miR-182-5p were enriched in the anti-Ago2 (a core component of the RNA-induced silencing complex) group. Moreover, the qRT-PCR results showed that miR-182-5p expression declined in HG-induced VSMCs compared to the NG group. The inhibitory effect of HG on the miR-182-5p expression could be reversed by si-hsa_circRNA_0008028 transfection and further promoted by the overexpression of hsa_circRNA_0008028 (Figure 3(d)). Altogether, hsa_circRNA_0008028 served as a miR-182-5p sponge and negatively regulated its expression.

### 3.4. miR-182-5p Inhibition Reverses the Effect of hsa_circRNA_0008028 Silence on HG-Stimulated VSMCs

As shown in Figure 4(a), the expression of miR-182-5p was significantly inhibited when transfected with miR-182-5p-inhibitor compared to the miR-NC group (Figure 4(a)). Subsequently, HG-stimulated VSMCs were transfected with si-hsa_circRNA_0008028 and/or miR-182-5p inhibitor. The miR-182-5p inhibitor also eliminated the si-hsa_circRNA_0008028 induced upregulation of miR-182-5p in HG-treated VSMCs (Figure 4(b)). Moreover, the suppressive effects of si-hsa_circRNA_0008028 on cell viability (Figure 4(c)), cell proliferation and cell cycle regulation (Figures 4(d) and 4(e)), ALP activity (Figure 4(f)), and osteoblast differentiation (Figure 4(g)) and autophagy (Figure 4(h)) in HG-treated VSMCs were all reversed by miR-182-5p inhibitor. The above evidence proved that hsa_circRNA_0008028 regulated HG-induced VSMC injury via miR-182-5p.

RETRACTED

### 3.5. TRIB3 Is a Downstream Target of miR-182-5p

Next, we further searched the downstream targets of miR-182-5p and predicted the binding sites between miR-182-5p and tribble 3 (TRIB3) 3′UTR region through TargetScan (Figure 5(a)). It was observed that the cotransfection of WT-TRIB3 3′UTR with miR-182-5p could significantly diminish the luciferase activity compared with the miR-NC group in VSMCs, while this inhibitory effect could be blocked in MUT-TRIB3 3′UTR transfected cells (Figure 5(b)). RIP assay also revealed that miR-182-5p and TRIB3 were specifically enriched in anti-Ago2 relative to the control anti-IgG group (Figure 5(c)), suggesting that TRIB3 served as a target of miR-182-5p. Moreover, the mRNA and protein expression of TRIB3 increased in the HG group compared with the NG group, and they both could be remarkably suppressed by miR-182-5p and promoted by miR-182-5p inhibitor in HG condition (Figures 5(d) and 5(e)).

### 3.6. TRIB3 Knockdown Blocks the Side Effects of HG on VSMCs

To explore the function of TRIB3 in HG-treated VSMCs, siRNA was used to interfere with TRIB3. The data verified that the HG condition promoted TRIB3 mRNA and protein expression, which was recovered and downregulated by si-TRIB3 transfection (Figure 6(a)). Subsequent results confirmed that interfering with TRIB3 could restore the accelerating effects of HG on VSMCs, including cell viability (Figure 6(b)), cell proliferation (Figures 6(c) and 6(d)), ALP activity (Figure 6(e)), osteoblast differentiation-related protein (Runx2, OPN, and *α*-SMA) expressions (Figure 6(f)), and autophagy-related protein (LC3B-II/LC3B-I and SQSTM1/p62) expressions (Figure 6(g)). Taken together, the knockout of TRIB3 weakened the HG-induced proliferation, calcification, and autophagy of VSMCs.

### 3.7. hsa_circRNA_0008028/miR-182-5p Regulates HG-Induced VSMC Dysfunctions through TRIB3

Ultimately, to identify the interactive associations among hsa_circRNA_0008028, miR-182-5p, and TRIB3 in VSMC proliferation, calcification, and autophagy, miR-182-5p inhibitor and/or si-hsa_circRNA_0008028 were used to transfect VSMCs. The TRIB3 levels were then detected by qRT-PCR and western blotting. The data showed that, compared to the NG group, TRIB3 expression level was increased when exposed to HG condition and was further promoted by miR-182-5p inhibitor but decreased by si-hsa_circRNA_0008028. At the same time, the effect of si-hsa_circRNA_0008028 on TRIB3 expression in HG-treated VSMCs was abolished by miR-182-5p inhibitor cotransfection (Figures 7(a) and 7(b)). These results indicated that TRIB3 was regulated by hsa_circRNA_0008028/miR-182-5p axis.

RETRACTED

Next, it was observed that miR-182-5p inhibitor enhanced cell proliferation and calcification, such as the upregulation of cell viability, ALP activity, and the protein expression of cyclin D1, Runx2, and OPN, while downregulated protein expression of *α*-SMA in VSMCs upon HG exposure, which was effectively reversed by si-hsa_circRNA_0008028 (Figures 7(c)–7(g)). Moreover, the increased LC3B-II/LC3B-I and the decreased SQSTM1/p62 induced by HG were strengthened by miR-182-5p inhibitor but weakened by si-hsa_circRNA_0008028 (Figure 7(h)). Nevertheless, the above effects were reversed when VSMCs were cocultured with si-hsa_circRNA_0008028 and miR-182-5p inhibitor (Figures 7(c)–7(h)). Thus, the results suggested that hsa_circRNA_0008028 knockdown attenuated HG-induced VSMC dysfunctions targeting miR-182-5p partly via TRIB3.

## 4. Discussion

In this study, it was revealed that HG could induce proliferation, calcification, and autophagy of VSMCs and identified that these effects were reversed by hsa_circRNA_0008028 deficiency or miR-182-5p overexpression. Mechanistically, it was first found that hsa_circRNA_0008028 could enhance the expression of TRIB3, a target gene of miR-182-5p as a miR-182-5p sponge. These findings provide new insight into noncoding RNAs in diabetic VSMC proliferation, calcification, and autophagy and indicate that modulation of the activity of noncoding RNAs, such as hsa_circRNA_0008028 and miR-182-5p, may become a novel therapeutic approach for diabetes-related vasculopathy.

Dysfunctions of VSMCs for the metabolism and phenotypic transformation are associated with the progression of vascular diseases, such as diabetes, pulmonary hypertension, and atherosclerosis [25]. In response to vascular injury, VSMCs dedifferentiate from a “contractile” phenotype to a “synthetic” phenotype, which features proliferation, migration, extracellular matrix (ECM) component production, and reduction of the VSMC-specific markers [25–28]. It was reported that hyperglycemia plays an important role in the pathogenesis of diabetes-related vascular diseases, including vascular calcification and atherosclerosis [29]. HG could promote proliferation and migration, induce oxidative stress and inflammation of VSMCs, and speed up the formation and accumulation of advanced glycation end products (AGEs), leading to vascular calcification [30–32]. In this study, EdU staining, as well as the increased cell viability, ALP activity, cell cycle, and osteogenic differentiation-related protein expression verified that VSMCs cultured in HG occurred in serious proliferation and calcification. Moreover, the upregulated LC3B-II/LC3B-I ratio and downregulated SQSTM1/p62 expression suggested that HG promoted the autophagy process of VSMCs. All in all, the data demonstrated that HG could promote the proliferation, calcification, and autophagy of VSMCs.

circRNAs, a type of noncoding RNAs without 3′- and 5′-ends, have been suggested to be a miRNA sponge to offset miRNA-mediated mRNA degradation, or a ceRNA to network with mRNA downstream of miRNA to regulate diverse biological processes [15, 33]. Recent evidence showed that some circRNAs and miRNAs got involved in the dysfunctions of VSMCs in HG conditions. For example, circRNA LRP6 promoted HG-induced phenotypic transformation of VSMCs by regulating the miR-545-3p/HMGA1 axis [2]. CircWDR77 silencing blocked the proliferation and migration of VSMCs by downregulating FGF2 expression via sponging miR-124 [15]. Besides, previous studies called that miR-504 promoted HG-induced VSMC dysfunction, and miR-145 protected against HG-induced VSMCs by suppressing ROCK1 [34, 35]. However, there are rare reports on the effect of hsa_circRNA_0008028 and its target miR-182-5p in the regulation of VSMC functions. In this study, it was found a circRNA, hsa_circRNA_0008028, was extensively expressed in HG-treated VSMCs, while its silencing induced by especial siRNAs resulted in a suppression of VSMC proliferation, calcification, and autophagy upon HG stimulation. Then, it was verified that miR-182-5p was a direct target of hsa_circRNA_0008028, and its inhibition could further promote VSMCs' dysfunction and weaken the protective effects of si-hsa_circRNA_0008028 on VSMCs exposed to HG. All in all, this study verified that hsa_circRNA_0008028 could sponge miR-182-5p in HG-treated VSMCs and its function in diabetic vasculopathy was associated with the regulation of miR-182-5p expression.

RETRACTED

As widely believed, miRNAs perform their functions by directly binding to their target mRNAs [36]. In this study, TRIB3, a 45 kDa pseudokinase identified as a target of miR-182-5p, was demonstrated to regulate metabolism and insulin signaling in diabetes-injured tissues, including liver, adipose tissue, heart, and skeletal muscle, and to be induced in a variety of cell types under different conditions of stress, including ER stress, nutrient deprivation, and oxidative stress [37–39]. Studies have shown that inhibiting the expression of TRIB3 can reduce vascular remodeling of VSMCs, but its regulating mechanism is still not very clear [19]. It was demonstrated that TRIB3 was a downstream target of miR-182-5p and significantly upregulated in VSMCs under HG conditions, and its knockdown reduced HG-induced proliferation, calcification, and autophagy of VSMCs. Moreover, its expression level and effects on HG-treated VSMCs were repressed by hsa_circRNA_0008028 knockout, which was offset by miR-182-5p inhibitor; that is, the regulatory role of hsa_circRNA_0008028/miR-182-5p in proliferation, calcification, and autophagy of VSMCs under HG condition was possibly achieved through TRIB3.

## 5. Conclusions

In conclusion, hsa_circRNA_0008028 was extensively expressed in HG-treated VSMCs in *vitro*, which can serve as the sponge of miR-182-5p and increase the expression of TRIB3, thus promoting HG-mediated proliferation, calcification, and autophagy of VSMCs. hsa_circRNA_0008028 is expected to be a molecular target for the diagnosis and treatment of diabetes-related vascular diseases.

## Figures and Tables

**Figure 1:** hsa_circRNA_0008028 is highly expressed in HG-treated VSMCs. (a) hsa_circRNA_000802 expression level detected by qRT-PCR. VSMCs were exposed to different concentrations of D-glucose (5.5, 10, 20, and 30 mmol/L) for 48 hours. MA was used as a negative control. ^∗∗^*p* < 0.05 vs. the 5.5 mmol/L group. (b) hsa_circRNA_000802 expression level in VSMCs under D-glucose (30 mmol/L) for 0, 12, 24, and 48 hours, respectively. ^∗∗^*p* < 0.05 vs. the 0 hour group. (c) Expression levels of hsa_circRNA_000802 and linear GAPDH were examined by qRT-PCR in VSMCs treated with RNase R^+^ or RNase R^–^. ^∗∗^*p* < 0.05.

**Figure 2:** Silencing hsa_circRNA_0008028 inhibits HG-induced proliferation, calcification, and autophagy of VSMCs. VSMCs were treated with normal D-glucose (NG, 5.5 mmol/L) or high D-glucose (HG, 30 mmol/L) and then transfected with siRNA negative control (HG + si-NC) or siRNA-hsa_circRNA_0008028 (HG+si-hsa_circRNA_0008028) for 48 hours. (a) The relative expression level of hsa_circRNA_000802 determined by qRT-PCR. (b) Cell viability measured by CCK-8. (c) Cell proliferation analysis measured by EdU staining. (d) Percentage of EdU positive cells. (e) ALP activity. (f) The protein expression of cyclin D1, Runx2, OPN, and *α*-SMA. (g) The protein expression of LC3B-II/LC3B-I and SQSTM1/p62. ^∗∗^*p* < 0.05 vs. the NG group; ^$$^*p* < 0.05 vs. the HG+si-NC group.

**Figure 3:** hsa_circRNA_0008028 binds to miR-182-5p. (a) Binding sites between hsa_circRNA_0008028 and miR-182-5p predicated using starBase. The mutated (Mut) version of hsa_circRNA_0008028 was shown. (b) Dual-luciferase reporter assay was used to verify the binding relationship between hsa_circRNA_0008028 and miR-182-5p. ^∗∗^*p* < 0.05 vs. the WT-hsa_circRNA_0008028 group. (c) RIP assay performed the endogenous correlation of hsa_circRNA_0008028 and miR-182-5p. ^∗∗^^or $$^*p* < 0.05 vs. the anti-IgG group. (d) qRT-PCR detected the miR-182-5p expression regulated by hsa_circRNA_0008028 silencing or over-expression. ^∗∗^*p* < 0.05 vs. the NG group; ^$$^*p* < 0.05 vs. the HG+si-NC group; ^##^*p* < 0.05 vs. the HG+Vector group.

**Figure 4:** miR-182-5p inhibition reverses the effect of hsa_circRNA_0008028 silence on HG-stimulated VSMCs. (a) qRT-PCR analysis of miR-182-5p expression transfected with miR-182-5p inhibitor. ^∗∗^*p* < 0.05 vs. the miR-NC group. (b–h) VSMCs were cotransfected with si-circ-hsa_circRNA_0008028 and/or miR-182-5p inhibitor and then subjected to HG stimulation. (b) miR-182-5p expression detected by qRT-PCR. (c) Cell viability analysis using CCK-8. (d) Cell proliferation analysis with EdU staining. (e) Percentage of EdU positive cells. (f) ALP activity. (g) Western blotting detection of cell cycle and osteogenic differentiation-related protein expression. (h) Western blotting examination of autophagy-related protein expression. ^∗∗^*p* < 0.05 vs. the NG group; ^$$^*p* < 0.05 vs. the HG+si-NC group; ^##^*p* < 0.05 vs. the HG +si-hsa_circ_00080+miR-NC group.

**Figure 5:** TRIB3 is a downstream target of miR-182-5p. (a) Binding sites between miR-182-5p and tribble 3 (TRIB3) 3′UTR predicated using the TargetScan software. The interaction between miR-182-5p and TRIB3 was measured by (b) dual luciferase reporter assay and (c) RIP assay. ^∗∗^^or $$^*p* < 0.05. (d) qRT-PCR and (e) western blotting detection of TRIB3 expression in VSMCs transfected with miR-NC, miR-182-5p, or miR-182-5p inhibitor and then exposed to HG. ^∗∗^*p* < 0.05 vs. the NG group; ^$$^*p* < 0.05 vs. the HG+miR-NC group.

**Figure 6:** TRIB3 knockdown blocks the side effects of HG on VSMCs. VSMCs were transfected with TRIB3 siRNA upon HG condition. (a) TRIB3 protein expression detected by western blotting. (b) Cell viability detection using CCK-8. (c) Cell proliferation observation by EdU staining. (d) Percentage of EdU positive cells. (e) ALP activity. (f) Western blotting detection of cell cycle and osteogenic differentiation-related protein expression. (g) Western blotting examination of autophagy-related protein expression. ^∗∗^*p* < 0.05 vs. the NG group; ^$$^*p* < 0.05 vs. the HG+si-NC group.

**Figure 7:** hsa_circRNA_0008028/miR-182-5p regulates HG-induced VSMC dysfunctions through TRIB3. VSMCs were transfected with si-circ-hsa_circRNA_0008028 and/or miR-182-5p inhibitor and then subjected to HG stimulation. The expression level of TRIB3 was detected by (a) qRT-PCR and (b) western blotting. (c) Cell viability reflection using CCK-8. (d) Cell proliferation examination using EdU staining. (e) Percentage of EdU positive cells. (f) ALP activity. The protein expression of (g) cyclin D1, Runx2, OPN and *α*-SMA, and (h) LC3B-II/LC3B-I and SQSTM1/p62 was detected by western blotting. ^∗∗^*p* < 0.05 vs. NG group; ^$$^*p* < 0.05 vs. the HG group; ^##^*p* < 0.05 vs. the HG+miR-182-5p inhibitor group; ^&&^*p* < 0.05 vs. the HG+si-hsa_circ_00080 group.

RETRACTED

## Data Availability

The data used to support the findings of this study are included within the article.

## Supplementary Materials

Supplementary Materials Table S1 shows the sequences of primers for qRT-PCR.
